# Association between oral health and cognitive function among Chinese older adults: the Taizhou imaging study

**DOI:** 10.1186/s12903-023-03353-9

**Published:** 2023-09-05

**Authors:** Wenjia Gu, Jialin Li, Fei Li, Teck-Ek Ho, Xiping Feng, Yingzhe Wang, Min Fan, Mei Cui, Kelin Xu, Xingdong Chen, Haixia Lu, Yanfeng Jiang

**Affiliations:** 1 Department of Preventive Dentistry, Shanghai Ninth People’s Hospital, College of Stomatology, National Center for Stomatology, Shanghai Key Laboratory of Stomatology, Shanghai Jiao Tong University School of Medicine, Shanghai Jiao Tong University, National Clinical Research Center for Oral Diseases, 639 Zhizaoju Road, Shanghai, 200011 China; 2 State Key Laboratory of Genetic Engineering, Human Phenome Institute, Zhangjiang Fudan International Innovation Center, Fudan University, Shanghai, China; 3 Fudan University Taizhou Institute of Health Sciences, Taizhou, Jiangsu China; 4 Department of Neurology, Huashan Hospital, Fudan University, Shanghai, China; 5 Taixing Disease Control and Prevention Center, Taizhou, Jiangsu China; 6 Department of Biostatistics, School of Public Health, Key Laboratory of Public Health Safety of Ministry of Education, Fudan University, Shanghai, China; 7 International Human Phenome Institute (Shanghai), Fudan University, 2005 Songhu Road, Shanghai, 200438 China

**Keywords:** Oral health, Dental caries, Periodontal status, Global cognition, Short-term memory, Executive function

## Abstract

**Background:**

We aimed to investigate the association between oral health and cognitive function in a sample of older adults from a Chinese rural community.

**Methods:**

The cross-sectional cognitive function of 677 individuals were assessed by Mini-Mental State Examination (MMSE) and Montreal Cognitive Assessment (MoCA). A comprehensive profile of the oral health status was evaluated by questionnaire and clinical examination.

**Results:**

Multiple covariates-adjusted regression models demonstrated decayed teeth (DT) and decayed/missing/filled teeth (DMFT) were negatively associated with MoCA score (all *p* < 0.05). Calculus index (CI) and clinical attachment loss (CAL) were significantly associated with the lower MoCA, short-term memory and executive function score, respectively (all *p* < 0.05). Additionally, participants with missing teeth unrestored tend to get lower MMSE and MoCA scores (*p* < 0.05). The results also showed that increased DT and CI were modestly associated with higher odds of cognitive impairment (*p* < 0.05).

**Conclusions:**

There is an association between oral health and global cognition. Poor periodontal status was strongly associated with worse global cognition performance, especially in the short-term memory and executive domain for the aging population.

**Supplementary Information:**

The online version contains supplementary material available at 10.1186/s12903-023-03353-9.

## Background

Oral health has become one of the most important concerned health problems in the world. Dental caries, periodontitis and other common oral diseases could cause tooth loss, thus affecting the quality of life. Globally, nearly half of the population suffered from oral diseases [1]. In China, it is estimated that the prevalence of dental caries is higher than 95% in the middle-aged and older population, while the periodontal health rate is merely less than 10% [2, 3]. Accumulating evidence has shown that poor oral health was significantly associated with higher incidence and prevalence of diseases, such as diabetes, cardiovascular disease, and gastrointestinal cancer, and is thus relevant to high mortality rates in older adults [4–9]. Overall, the generally poor oral hygiene of older adults has prompted increasing concern about the impact of oral disease on their health, such as debilitation and cognitive decline [10].

Cognitive impairment is a common chronic disease among older adults worldwide, which seriously affects their daily life and social competence [11]. China has the highest number of people with cognitive impairment in the world, and accounts for approximately a quarter of the entire dementia cases worldwide [12]. Considering the irreversible progression and uncertain therapies of dementia, identifying and intervening in modifiable risk factors is crucial for disease prevention and control [13]. The Lancet Commission has reported that controlling 12 modifiable risk factors, such as smoking, obesity, depression, and alcohol consumption, can delay and prevent approximately 40% of dementia cases worldwide [14]. Recently, an exposure-wide association study also indicated that multiple lifestyles and medical history, including dental health, were potential targets for the prevention of dementia [15]. However, as a promising modifiable factor, the association between poor oral health status and dementia remains controversial. Previous studies have explored the relationship between oral health and cognitive function but have not reached a consistent conclusion [10, 16]. Most studies conducted in Western populations, focusing merely on tooth loss as an indicator of oral health [10, 17]. Therefore, given the variations in oral habits and dementia prevalence among different populations, it is urgent to detailed investigate the associations of oral health with dementia in more community-based populations.

Based on the Taizhou Imaging Study (TIS), we comprehensively assessed the oral health status by incorporating detailed questionnaires on oral hygiene habits and clinical oral examinations, including assessment of dental caries, periodontal conditions, and restoration of missing teeth. Furthermore, this study aims to explore the association between oral health and cognitive function, as well as dementia, providing additional evidence to enhance our understanding of this relationship.

## Methods

### Study design and participants

The TIS is an ongoing community-based cohort nested in the Taizhou Longitudinal Study, which aims to investigate lifestyle factors, multi-omics features, and age-related diseases in rural older Chinese. The rationale, aims, study design, and organization of TIS have been detailed previously [18]. Epidemiological questionnaire survey, physical and clinical examination, and biospecimen collection were conducted during the baseline (from 2013 to 2018) and subsequent follow-up visits, while oral examination began during the second round of follow-ups in 2020. In brief, a total of 904 individuals aged 55–65 years without a history of physician-diagnosed stroke, dementia, cancer, and other severe diseases were enrolled at baseline and 704 of them finished the follow-up survey in 2020. Participants without oral examination were further excluded (N = 27), leaving 677 participants as the final analysis set in this study. The TIS was approved by the Ethics Committee of the School of Life Sciences, Fudan University and Fudan University Taizhou Institute of Health Sciences (institutional review board approval number: 496 and B017, respectively). Written informed consent was obtained from each participant before enrollment and data collection.

### Cognitive function assessment

Global cognition is a summary of various cognitive domains such as attention and execution, assessed by the Chinese version of Mini-Mental State Examination (CMMSE) and the Beijing version of Montreal Cognitive Assessment (MoCA-BJ) in this study [19]. These two instruments have been linguistically and culturally adapted separately from the original English version and have both been tested in Chinese populations to ensure excellent reliability and validity [20, 21]. As proposed by Nasreddine, the MoCA was divided into six cognitive domains, including short-term memory (5 points), visuospatial abilities (4 points), executive functions (4 points), attention, concentration, and working memory (6 points), language (5 points) and orientation (6 points) [22].

Cognitive assessment was conducted in separate rooms to avoid learning effects between participants. An expert committee of neurologists and neuropsychologists adjudicated and reached consensus on the diagnosis of mild cognitive impairment (MCI) and dementia according to the Diagnostic and Statistical Manual of Mental Disorders, 4th edition (DSM-IV) criteria. According to the criteria suggested by Petersen, only those participants without dementia were given a diagnosis of MCI [23].

### Oral health assessment

Oral-related behaviors such as the number of missing teeth and toothbrushing daily frequency (0–1 time or 2–3 times), of each participant were obtained through an interviewer-administered questionnaire. Clinical oral examination was performed by two professional dentists, mainly included dental caries, periodontal status, and restoration of missing teeth.

According to the WHO’s criteria, dental caries condition examination was carried out by visual inspection combined with probing using a Community Periodontal Index (CPI) probe under artificial light [24]. Coronal and root dental caries of the entire mouth were examined, including the third molar. Decayed teeth (DT), missing teeth (MT), filled teeth (FT) due to coronal caries were recorded separately, coronal caries experience was also rating by the decayed/missing/filled teeth (DMFT) score, which was calculated by counting the number of DT, MT and FT. The decayed and filled root (DFRoot) score was generated by counting the number of decayed (D) and filled (F) root due to root surface caries. Root fragments were grouped in DT.

The periodontal clinical examination was performed using a periodontal probe (PCPUNC15, Hu-Friedy, Chicago, IL, USA) and a CPI probe, including Gingival bleeding index (GBI), Calculus index (CI), Probing depth (PD), and Clinical attachment loss (CAL) [24, 25]. First, CI of each tooth was obtained by visually examination in the whole mouth and subgingival calculus was not assessed. Then, a completely randomized method was used to randomly divide the subjects into two groups to receive quadrant I and III half-mouth examinations or quadrant II and IV half-mouth examinations of GBI, PD, CAL. This method can be used as an alternative to a full-mouth periodontal examination in population-based study with high accuracy [26]. For the GBI and CI, we examined the labial (buccal) and lingual (palatal) surfaces per tooth, and for the PD and CAL, six sites (mesio-buccal, mid-buccal, disto-buccal, mesio-lingual, mid-lingual, and disto-lingual) per tooth were examined. Whether the missing teeth had been restored was also recorded.

The calibration session was conducted between the two physicians that performed the oral clinical examination. Firstly, the training of all indices was conducted. After training, each physician practiced the examination on a group of 10 participants in the outpatient service of Shanghai Ninth people’s hospital. Then two physicians independently examine the same group of 20 participants and compare his or her findings with another physician. If there are major discrepancies, the participants should be re-examined so that inter-examiner differences can be reviewed and resolved by group discussion. The calibration was continued until the high level of consistency of physician was achieved. During the implementation of oral clinical examination, participants were randomly assigned to one of the two physicians for oral clinical examination. Approximately 10% of these participants were re-examined to monitor inter-examiner reproducibility. As measured using intraclass correlation coefficient (ICC) statistics, the inter-examiner reliabilities of DMFT, DFRoot, CI, GBI, PD, and CAL were 0.97, 0.75, 0.92, 0.60, 0.77, and 0.75, respectively.

### Diagnosis of periodontitis

Periodontitis was diagnosed according to the criteria for periodontitis grading updated by the Centers for Disease Control and Prevention and the American Academy of Periodontology (CDC/AAP criteria) in 2012 [27]. This criteria showed high agreement with the European Federation Periodontology and the American Academy of Periodontology (EFP/AAP criteria) in 2018, especially in a rural sample with high periodontitis occurrence [28, 29]. As this study adopted half-mouth examinations, periodontitis was defined according to a half-reduced CDC/AAP definition: (1) mild periodontitis: ≥1 interproximal sites with CAL ≥ 3 mm, along with ≥ 1 interproximal sites PD ≥ 4 mm; (2) moderate periodontitis: ≥1 interproximal sites CAL ≥ 4 mm, or ≥ 1 interproximal sites PD ≥ 5 mm; (3) severe periodontitis: ≥1 interproximal sites (not the same tooth) CAL ≥ 6 mm, along with ≥ 1 interproximal sites PD ≥ 5 mm [30, 31]. Complete edentulism was classified as severe periodontitis.

### Covariates

Information on demographics (age, sex, years of education, etc.), lifestyle (current smoking, alcohol consumption, etc.), socioeconomic status, and medical history was collected by a standardized questionnaire administered by trained interviewers [18]. Medical history of hypertension, diabetes, and hyperlipidemia were obtained from physicians’ diagnosis and physical examination. Anthropometry was examined in-person by experienced technicians, and body mass index (BMI, kg/m^2^) was calculated according to height and weight.

### Statistical analysis

For basic demographic information and oral health indicators, continuous variables were described by median (P_25_, P_75_) due to the abnormal distribution, and categorical variables were presented as frequencies (%). The Mann-Whitney U test was conducted for continuous variables and the chi-square test was used for categorical variables to test the differences between groups. The Spearman rank correlation test was used to calculate the correlation of global cognition scores with continuous demographics variables and oral health indicators.

Considering that the MMSE and MoCA scores are bounded continuous variables ([0,30] score), it was difficult to find a suitable method to convert them into a normal distributed data form. Therefore, the MMSE and MoCA scores were transformed into variables conforming to a beta distribution with an open interval of (0, 1), and beta regression was selected to analyze the association between oral health indicators and global cognition scores [32–34]. As the scores for the cognitive domains were integers ranging from 0 to 6, which were count variables, Poisson regression was applied to evaluate the association between oral health and six cognitive domain scores [35]. In exploring the association between oral health and cognitive impairment, the outcome was the presence or absence of cognitive impairment (MCI and dementia), which was a dichotomous variable, so multifactor logistic regression was conducted [36]. Considering the number of dementia group was relatively small (N = 55), the MCI and dementia groups were combined as cognitive impairment group, and multiple logistic regression was further performed. All estimates were calculated in units of per standard deviation (SD) increase for continuous oral health indicators in regression models. Two models were developed for all multivariate analyses: model 1 was adjusted for age, sex, and years of education, and model 2 was further adjusted for toothbrushing frequency, smoking, alcohol consumption, hypertension, diabetes, and hyperlipidemia. All analyses were performed in R (version 4.1.0). Differences were considered to be statistically significant at *p* < 0.05.

## Results

### Characteristics of the study participants

Table 1 shows the selected characteristics of the study participants (N = 677, male:43.7%, female:56.3%). Males had a significantly lower BMI and lower rates in hyperlipidemia, whereas higher rates of smoking and alcohol consumption than those in female (all *p* < 0.05). The prevalence of dementia and MCI was 8.1% and 27.6% respectively. The MMSE and MoCA scores and the proportion of cognitively normal were significantly higher in males than in females (all *p* < 0.001). The mean DMFT in the study population was 8.4, and the prevalence of severe periodontitis (including complete edentulism) was 52.9%. The number of participants without or with mild periodontitis was seven, thus combined with moderate group and showed in Table 1. DT and DMFT were significantly higher in female, while CI, CAL, and the proportion of severe periodontitis were significantly higher in male (all *p* < 0.05). This indicated that females suffered more dental caries, while males had worse periodontal status. The correlation between characteristics of the study population and the MMSE and MoCA scores is presented in Table 1.

**Table 1:** Demographics, oral health, and cognition of the study participants

Variables		Total (N = 677)	Male (N = 296)	Female (N = 381)	*p* value
Age (years)		66.0 (63.0, 68.0)	66.0 (63.0, 68.0)	65.0 (63.0, 67.0)	0.382
BMI (kg/m^2^)		23.1 (20.9, 25.3)	22.4 (20.4, 24.8)	23.3 (21.6, 25.7)	**< 0.001**
Education (year)		5.0 (0.0, 9.0)	9.0 (6.0, 9.0)	1.0 (0.0, 6.0)	**< 0.001**
Toothbrushing frequency					0.134
	0–1 time daily	404 (59.7)	180 (60.8)	224 (58.8)	
	2–3 times daily	141 (20.8)	52 (17.6)	89 (23.4)	
	Missing	132 (19.5)	64 (21.6)	68 (17.9)	
Smoking		231 (34.1)	223 (75.3)	8 (2.1)	**< 0.001**
Alcohol consumption		241 (35.6)	212 (71.6)	29 (7.6)	**< 0.001**
Hypertension		273 (40.3)	108 (36.5)	165 (43.3)	0.086
Diabetes		70 (10.3)	26 (8.8)	44 (11.6)	0.296
Hyperlipidemia		325 (48.0)	121 (40.9)	204 (53.5)	**0.001**
MMSE		25 (21, 27)	27 (24, 28)	23 (17, 26)	**< 0.001**
MoCA		16 (12, 21)	19 (16, 23)	13 (9, 18)	**< 0.001**
Cognitive group					**< 0.001**
	Normal cognition	435 (64.3)	216 (73.0)	219 (57.5)	
	MCI	187 (27.6)	75 (25.3)	112 (29.4)	
	Dementia	55 (8.1)	5 (1.7)	50 (13.1)	
DT		2.5 (3.2)	2.0 (2.6)	3.0 (3.4)	**< 0.001**
MT		5.7 (6.1)	5.3 (5.6)	6.1 (6.5)	0.091
FT^*^		0.1 (0.4)	0.1 (0.3)	0.1 (0.5)	0.174
DMFT		8.4 (7.1)	7.3 (6.6)	9.2 (7.4)	**< 0.001**
DFRoot		0.6 (1.2)	0.6 (1.1)	0.7 (1.3)	0.339
Present tooth number		26.3 (6.1)	26.7 (5.6)	26.0 (6.5)	0.091
CI		0.7 (0.2)	0.7 (0.2)	0.6 (0.2)	**< 0.001**
GBI		0.4 (0.3)	0.4 (0.3)	0.4 (0.3)	0.591
PD, mm		1.8 (0.6)	1.8 (0.6)	1.8 (0.6)	0.091
CAL, mm		3.2 (1.1)	3.4 (1.2)	3.0 (1.0)	**< 0.001**
Severity of periodontitis (%)					**0.044**
	No/Mild/Moderate	319 (47.1)	126 (42.6)	193 (50.7)	
	Severe or edentulous	358 (52.9)	170 (57.4)	188 (49.3)	
Restoration of missing teeth (%)					0.434
	No missing teeth unrestored	374 (55.2)	158 (53.4)	216 (56.7)	
	With missing teeth unrestored	303 (44.8)	138 (46.6)	165 (43.3)	

Data were presented as N (%) or median (P_25_, P_75_) or mean (SD).

Abbreviation: BMI, body mass index; CAL, clinical attachment loss; CI, calculus index; DFRoot, decayed and filled root; DMFT, decayed, missing and filled teeth; DT, decayed teeth; FT, filled teeth; GBI, gingival bleeding index; MCI, mild cognitive impairment; MMSE, Mini-Mental State Examination; MoCA, Montreal Cognitive Assessment; MT, missing teeth; PD, probing depth

The Mann-Whitney U test and the chi-square test were used to calculate *p* values

### Association between oral health and global cognition

The correlation between oral health and cognitive function is displayed in **sTable 2**. The MMSE and MoCA scores were negatively correlated with DT (ρ = -0.16, *p* < 0.001; ρ = -0.17, *p* < 0.001), DMFT (ρ = -0.15, *p* < 0.001; ρ = -0.18, *p* < 0.001), and GBI (ρ = -0.09, *p* = 0.017; ρ = -0.14, *p* < 0.001). Similarly, MT was inversely correlated with global cognition (MMSE: ρ = -0.07, *p* = 0.080; MoCA: ρ = -0.11, *p* = 0.004). Nevertheless, FT, DFRoot, CI, PD, CAL, severity of periodontitis, and restoration of missing teeth had no statistically significant correlation with the MMSE and MoCA scores (all *p* > 0.05).

Multivariate analyses were conducted to further investigate the associations between oral health and global cognition, indicated by the MMSE and MoCA scores (Table 2). Results showed that FT, DMFT, and CI had modest associations with decreased MMSE score (regression coefficients: -0.08, -0.07 and − 0.10, respectively, all *p* < 0.05 in model 1). In terms of the MoCA score, significant associations were found with DT, DMFT, CI, and CAL (regression coefficients range from − 0.11 to -0.05, all *p* < 0.05 in both two models). Restoration of missing teeth negatively associated with the MMSE and MoCA score only in model 2 (regression coefficient = -0.15, *p* = 0.038; regression coefficient = -0.12, *p* = 0.035).

**Table 2:** The associations between oral health and global cognition

Oral health	Model	MMSE score			MoCA score		
		Coefficient	SE	*p* value	Coefficient	SE	*p* value
DT	1	-0.05	0.03	0.149	-0.08	0.03	**0.002**
	2	-0.07	0.03	0.050	-0.09	0.03	**0.001**
MT	1	-0.05	0.03	0.140	-0.05	0.03	0.054
	2	-0.01	0.04	0.782	-0.04	0.03	0.190
FT	1	-0.08	0.03	**0.011**	0.00	0.02	0.979
	2	-0.05	0.04	0.152	0.03	0.03	0.306
DMFT	1	-0.07	0.03	**0.039**	-0.08	0.03	**0.001**
	2	-0.04	0.04	0.225	-0.08	0.03	**0.004**
DFRoot	1	-0.01	0.03	0.820	-0.03	0.03	0.214
	2	-0.03	0.03	0.445	-0.05	0.03	0.081
CI	1	-0.10	0.03	**0.002**	-0.11	0.03	**< 0.001**
	2	-0.07	0.04	0.051	-0.11	0.03	**< 0.001**
GBI	1	0.01	0.03	0.852	-0.02	0.03	0.394
	2	-0.01	0.03	0.764	-0.03	0.03	0.271
PD	1	0.04	0.03	0.173	0.02	0.03	0.549
	2	0.01	0.03	0.801	0.00	0.03	0.862
CAL	1	-0.02	0.03	0.542	-0.05	0.03	**0.033**
	2	-0.02	0.03	0.514	-0.07	0.03	**0.008**
Severity of periodontitis	1	0.03	0.07	0.621	-0.03	0.05	0.511
	2	0.04	0.07	0.570	-0.07	0.05	0.187
Restoration of missing teeth	1	-0.04	0.07	0.495	-0.05	0.05	0.280
	2	-0.15	0.07	**0.038**	-0.12	0.05	**0.035**

Abbreviation: CAL, clinical attachment loss; CI, calculus index; DFRoot, decayed and filled root; DMFT, decayed, missing and filled teeth; DT, decayed teeth; FT, filled teeth; GBI, gingival bleeding index; MMSE, Mini-Mental State Examination; MoCA, Montreal Cognitive Assessment; MT, missing teeth; PD, probing depth; SE, standard error

Model 1 was adjusted for age, sex, and years of education. Model 2 was further adjusted for toothbrushing frequency, smoking, alcohol consumption, hypertension, diabetes, and hyperlipidemia

### Associations between oral health and cognitive domain scores

We additionally assessed the associations between oral health indicators and six cognitive domain scores derived from MoCA. We found that CI and CAL were significantly associated with short-term memory and executive function (Table 3). In the fully adjusted model 2, per-SD increase in CI and CAL was separately associated with a 14% and 16% decrease (95% confidence interval: 5-22% and 7-25%, respectively) in short-term memory score. Similarly, per-SD increase in CI and CAL was separately associated with a 9% and 7% decrease (95% confidence interval: 3-14% and 1-13%, respectively) in executive function score. Visuospatial and orientation domain were negatively associated with CI only in model 1. Generally, oral health had a strong associated with short-term memory and executive function, while the associations with the other cognitive domain scores were modest or non-significant after covariates adjustment, including visuospatial abilities attention/concentration/working memory, language, and orientation (**sTable 3**).

**Table 3:** The associations of oral health with short-term memory and executive function

Oral health	Model	short-term memory		executive function	
		exp(coef)	95%CI	exp(coef)	95%CI
DT	1	0.94	(0.85, 1.04)	0.99	(0.93, 1.05)
	2	0.91	(0.81, 1.02)	0.99	(0.92, 1.05)
MT	1	0.92	(0.83, 1.02)	0.96	(0.90, 1.02)
	2	0.94	(0.83, 1.04)	0.96	(0.90, 1.03)
FT	1	1.00	(0.91, 1.09)	1.02	(0.96, 1.07)
	2	1.00	(0.89, 1.10)	1.01	(0.95, 1.07)
DMFT	1	0.91	(0.82, 1.01)	0.96	(0.90, 1.02)
	2	0.91	(0.81, 1.01)	0.96	(0.90, 1.03)
DFRoot	1	0.96	(0.87, 1.06)	1.01	(0.95, 1.07)
	2	0.92	(0.82, 1.02)	0.99	(0.93, 1.06)
CI	1	**0.88**	**(0.80, 0.96)**	**0.93**	**(0.88, 0.98)**
	2	**0.86**	**(0.78, 0.95)**	**0.91**	**(0.86, 0.97)**
GBI	1	0.92	(0.83, 1.00)	0.98	(0.93, 1.04)
	2	0.93	(0.84, 1.02)	0.97	(0.91, 1.03)
PD	1	0.97	(0.88, 1.06)	0.99	(0.94, 1.04)
	2	0.94	(0.85, 1.04)	0.97	(0.92, 1.03)
CAL	1	**0.86**	**(0.78, 0.95)**	0.95	(0.89, 1.00)
	2	**0.84**	**(0.75, 0.93)**	**0.93**	**(0.87, 0.99)**
Severity of periodontitis	1	0.87	(0.72, 1.04)	1.03	(0.92, 1.14)
	2	0.88	(0.72, 1.07)	1.01	(0.90, 1.14)
Restoration of missing teeth	1	0.85	(0.70, 1.02)	1.06	(0.95, 1.18)
	2	0.84	(0.68, 1.02)	1.07	(0.94, 1.20)

Abbreviation: 95%CI, 95% confidence interval; CAL, clinical attachment loss; CI, calculus index; DFRoot, decayed and filled root; DMFT, decayed, missing and filled teeth; DT, decayed teeth; exp(coef), exponential coefficient; FT, filled teeth; GBI, gingival bleeding index; MT, missing teeth; PD, probing depth

Model 1 was adjusted for age, sex, and years of education. Model 2 was further adjusted for toothbrushing frequency, smoking, alcohol consumption, hypertension, diabetes, and hyperlipidemia

### Association between oral health and cognitive impairment

Table 4 shows multiple logistic regression of oral health with cognitive impairment. Each SD increase in DT and CI were associated with higher odds ratio (OR) of cognitive impairment in model 1 (OR and 95% confidence interval: 1.20 (1.01, 1.41) and 1.24 (1.04, 1.48), respectively). However, no significant associations were found between oral health and cognitive impairment in model 2. When specifically differentiated between MCI and dementia, the associations of cognitive impairment with DT and CI were modest or nonsignificant (*p* ≤ 0.05).

**Table 4:** The associations between oral health and cognitive impairment (OR (95%CI)).

Oral health	Model	Cognitive impairment	MCI	Dementia
DT	1	**1.20 (1.01, 1.41)**	1.16 (0.96, 1.38)	1.32 (1.00, 1.75)
	2	1.09 (0.90, 1.31)	1.00 (0.81, 1.23)	1.42 (1.01, 2.04)
MT	1	1.03 (0.88, 1.21)	1.04 (0.87, 1.24)	1.00 (0.73, 1.32)
	2	0.96 (0.79, 1.15)	0.96 (0.78, 1.17)	0.99 (0.63, 1.49)
FT	1	0.96 (0.81, 1.13)	0.92 (0.74, 1.11)	1.11 (0.82, 1.41)
	2	0.94 (0.75, 1.14)	0.92 (0.71, 1.13)	1.01 (0.66, 1.39)
DMFT	1	1.11 (0.94, 1.31)	1.10 (0.92, 1.31)	1.15 (0.86, 1.54)
	2	1.00 (0.82, 1.20)	0.96 (0.78, 1.17)	1.24 (0.83, 1.85)
DFRoot	1	0.99 (0.84, 1.16)	0.97 (0.81, 1.16)	1.00 (0.75, 1.30)
	2	0.98 (0.82, 1.17)	0.95 (0.77, 1.15)	1.05 (0.77, 1.43)
CI	1	**1.24 (1.04, 1.48)**	**1.20 (1.00, 1.45)**	1.36 (0.98, 1.94)
	2	1.22 (1.00, 1.48)	1.21 (0.99, 1.49)	1.31 (0.86, 2.04)
GBI	1	0.97 (0.82, 1.15)	0.98 (0.82, 1.17)	0.92 (0.68, 1.25)
	2	1.00 (0.83, 1.21)	0.99 (0.81, 1.21)	0.98 (0.68, 1.41)
PD	1	0.98 (0.83, 1.16)	1.02 (0.86, 1.21)	0.79 (0.53, 1.13)
	2	1.04 (0.86, 1.25)	1.07 (0.88, 1.29)	0.97 (0.60, 1.51)
CAL	1	1.06 (0.89, 1.25)	1.09 (0.92, 1.29)	0.87 (0.60, 1.22)
	2	1.08 (0.90, 1.29)	1.11 (0.92, 1.33)	0.98 (0.61, 1.51)
Severity of periodontitis	1	0.79 (0.57, 1.10)	0.80 (0.56, 1.14)	0.70 (0.37, 1.30)
	2	0.89 (0.61, 1.30)	0.87 (0.58, 1.30)	0.86 (0.40, 1.83)
Restoration of missing teeth	1	1.06 (0.76, 1.47)	1.11 (0.78, 1.57)	0.80 (0.42, 1.50)
	2	1.11 (0.76, 1.62)	1.05 (0.70, 1.57)	1.22 (0.56, 2.67)

Abbreviation: 95%CI, 95% confidence interval; CAL, clinical attachment loss; CI, calculus index; DFRoot, decayed and filled root; DMFT, decayed, missing and filled teeth; DT, decayed teeth; FT, filled teeth; GBI, gingival bleeding index; MCI, mild cognitive impairment; MT, missing teeth; OR, odds ratio; PD, probing depth

Cognitive impairment included MCI and dementia

Model 1 was adjusted for age, sex, and years of education. Model 2 was further adjusted for toothbrushing frequency, smoking, alcohol consumption, hypertension, diabetes, and hyperlipidemia

## Discussion

We performed a cross-sectional study to investigate the relationship between oral health and cognitive function in rural Chinese older adults. Some of oral health indicators, including DT, DMFT, and CI, were negatively correlated with global cognition. In addition, CI and CAL were significantly associated with short-term memory and executive function. DT and CI were associated with greater odds ratio of cognitive impairment. Dementia is a continuum lasting 15–25 years, and impairment in one or more cognitive domains is an essential prodromal stage preceding clinical dementia [37, 38]. Our study was based on a community population, the majority of whom were in a normal cognitive state or at a preclinical stage of dementia, suggesting the cognitive domain may more sensitive than global cognition to indicating cognitive impairment. Although the underlying mechanism of the association between cognitive domains and oral health remains unclear, it is of great significance to explore the risk factors of domain-specific cognitive function. The detailed investigation revealed the cognitive domains most closely associated with oral health, which expanding our understanding of the association.

In this study, the mean DT and DMFT were found to be significantly associated with global cognition and cognitive impairment, which was similar with previous studies. For instance, systematic reviews presented that people with dementia were more likely to develop coronal dental caries compared to non-demented people [16, 39]. A study conducted in older adults in Hong Kong (China) showed that after matching for gender and age, the mean DMFT was higher and statistically significant in the demented group than in the non-demented group [40]. These results suggest there might be a link between coronal dental caries and cognitive function. However, no clear biological mechanism for cognitive impairment causing caries has been found. It has been shown that with good dental care, the dental status of patients with dementia is not significantly different from that of patients without dementia [41, 42]. Therefore, at present, we consider that cognitive impairment leads to caries mainly due to behavioral changes, such as reduced ability of oral self-care and change in dietary habits [43, 44]. On the other hand, with the development of dental caries, microbial diversity decreased and the concentration of some neuroinflammatory markers would increase, which might promote the occurrence of cognitive dysfunction [45]. Although previous studies showed that root dental caries was more prevalent in dementia cases [39], we didn’t find any significant association of root dental caries and cognitive function, similar to the result of a previous study [46]. It could be ascribed to the high proportion of retained and unexposed roots in our study population, resulting in a low mean value of DFRoot, thus partly masking the relationship between root dental caries and cognitive function.

In terms of periodontal status, we collected GBI, CI, PD and CAL indexes. Plaque biofilm is the initiator of periodontal disease and calculus is formed when plaque calcify. Due to the prevailing subpar oral hygiene within the study population, a majority exhibited plaque on virtually all tooth surfaces. Moreover, the presence of calculus on specific tooth surfaces differed across individuals. As a result of these considerations, we ultimately opted for the CI for our analysis. This study found that CI was weakly associated with the MMSE score and cognitive impairment. In contrast, some studies revealed that the MMSE was related to PD, CAL, and periodontitis severity [47–49]. The high prevalence and severity of periodontitis in this study population resulted in minimal difference in periodontitis severity, which might obscure the relationship between periodontal status and cognitive function. In addition, most participants had severe gingival recession, and thus generally had a small PD. It might account for the lack of significant differences in PD between those with different cognitive status. In present study, those with lower MoCA score had higher CI and CAL, mainly reflected in short-term memory and executive capacity. It is a common conclusion that cognitive function was poorer in those with poor periodontal status. In addition to weakened awareness of oral health care, the possible mechanisms by which periodontal status affects cognitive function include direct process through blood flow, indirect process through inflammatory mediators, and induction of platelet aggregation protein expression [45, 50].

As a phenotype of masticatory performance, we also evaluated the restoration of missing teeth of each participant and found it was significantly associated with worse global cognition, short-term memory and executive performance. Similarly, a study indicated that residents with dentures had significantly higher cognitive score (MMSE) compared to edentulous adults without dentures [51]. It suggested that maintenance and adequate restoration of the masticatory system were important to prevent cognitive decline. Reduced masticatory function leads to a decrease in the release of specific mediators from the masticatory muscles, as well as an inadequate access to blood flow, both of which play a role in cognitive degeneration [52].

The major strength of this study is that we did a detailed oral examination, involving coronal dental caries, root dental caries, number of missing teeth, periodontal clinical indicators, and restoration of missing teeth. There are several limitations should be acknowledged. First, it was a cross-sectional study and the causal relationship between oral health and cognitive function could not be determined. Therefore, further longitudinal studies of the population and laboratory analyses of dental plaque and gingival sulcus samples are warranted. Secondly, the questionnaire did not include inquiries about the participants’ history of periodontal treatment, which might potentially affect the diagnosis of periodontitis and the evaluation of relevant parameters. In subsequent follow-up assessments, the questionnaire will incorporate a section to capture the history of periodontal treatment. In addition, further research is needed on the possible mechanisms underlying the association of periodontal status with short-term memory and executive capacity.

## Conclusion

In conclusion, there is an association between oral health and global cognition. Poor periodontal status was strongly associated with worse global cognition performance, especially in the short-term memory and executive domain for the aging population.

### Electronic supplementary material

Below is the link to the electronic supplementary material.

Supplementary Material 1

## Data Availability

The data analyzed in this study were obtained from the Taizhou Imaging Study. Further enquiries can be directed to the corresponding author.

## List of abbreviations

BMI: Body mass index
CAL: Clinical attachment loss
CDC/AAP: Centers for Disease Control and Prevention and the American Academy of Periodontology
CI: Calculus index
CPI: Community Periodontal Index
DFRoot: Decayed and filled root
DMFT: Decayed, missing and filled teeth
DSM-IV: Diagnostic and Statistical Manual of Mental Disorders, 4th edition
DT: Decayed teeth
EFP/AAP: European Federation Periodontology and the American Academy of Periodontology
FT: Filled teeth
GBI: Gingival bleeding index
ICC: Intraclass correlation coefficient
MCI: Mild cognitive impairment
MMSE: Mini-Mental State Examination
MoCA: Montreal Cognitive Assessment
MT: Missing teeth
PD: Probing depth
SD: Standard deviation
TIS: Taizhou Imaging Study
